# A Computational Framework to Identify Transcriptional and Network Differences between Hepatocellular Carcinoma and Normal Liver Tissue and Their Applications in Repositioning Drugs

This article has been retracted.

**DOI:** 10.1155/2021/9921195

**Published:** 2021-09-23

**Authors:** Aimin Hu, Zheng Wei, Zuxiang Zheng, Bichao Luo, Jieming Yi, Xinhong Zhou, Changjiang Zeng

**Affiliations:** Xiantao First People's Hospital Affiliated to Yangtze University, Xiantao 433000, China

## Abstract

Hepatocellular carcinoma (HCC) is one of the most common and lethal malignancies worldwide. Although there have been extensive studies on the molecular mechanisms of its carcinogenesis, FDA-approved drugs for HCC are rare. Side effects, development time, and cost of these drugs are the major bottlenecks, which can be partially overcome by drug repositioning. In this study, we developed a computational framework to study the mechanisms of HCC carcinogenesis, in which drug perturbation-induced gene expression signatures were utilized for repositioning of potential drugs. Specifically, we first performed differential expression analysis and coexpression network module analysis on the HCC dataset from The Cancer Genome Atlas database. Differential gene expression analysis identified 1,337 differentially expressed genes between HCC and adjacent normal tissues, which were significantly enriched in functions related to various pathways, including *α*-adrenergic receptor activity pathway and epinephrine binding pathway. Weighted gene correlation network analysis (WGCNA) suggested that the number of coexpression modules was higher in HCC tissues than in normal tissues. Finally, by correlating differentially expressed genes with drug perturbation-related signatures, we prioritized a few potential drugs, including nutlin and eribulin, for the treatment of hepatocellular carcinoma. The drugs have been reported by a few experimental studies to be effective in killing cancer cells.

## 1. Introduction

Liver cancer was the fifth most common cancer in 2012, accounting for 9.1% of global cancer deaths [1]. Most liver cancers (83%) are diagnosed in less developed countries, mainly in Asia, Africa, and Southern Europe. The vast majority (75%-90%) of primary liver cancers are hepatocellular carcinomas (HCCs), the most common and deadly malignant tumor worldwide [2, 3]. HCC usually occurs in cases with liver cirrhosis caused by viral infection and chronic inflammatory liver disease caused by exposure to chemical carcinogens. Known risk factors for HCC include chronic hepatitis B virus (HBV) and hepatitis C virus (HCV) infection, dietary aflatoxin exposure, fatty liver disease, alcoholic cirrhosis, obesity, smoking, diabetes, and iron overload [4, 5]. Patients are often diagnosed at advanced stages of liver cancer, and chemotherapy and immunotherapy are the most feasible treatment options.

Unfortunately, despite extensive research on the molecular mechanism of liver carcinogenesis, there are still only a few effective treatment options. Very little is known about the pathogenesis of most types of cancers, including liver cancer [6–8]. In the past few decades, about 130-180 anticancer drugs have been approved by the US FDA for use in clinical treatment [9]. Despite the increasing research on cancer drugs using model species (supported by nonhuman data) and nearly 1,000 drugs having been formulated using combinations of FDA-approved anticancer drugs, there is still uncertainty about the efficacy of these drugs in the treatment of cancer due to insufficient understanding of the molecular mechanisms of the disease [10–13]. This uncertainty poses the challenge of expensive clinical trials for the pharmaceutical industry. Thus, research and development of new drugs for the treatment of cancer and rational use of such drugs are still a big scientific issue. An alternative way is to perform drug repositioning, that is, identifying novel usage of existing drugs. Drug repositioning has been widely used in cancers [14–16] and other diseases including the recent outbreaking COVID-19 [17, 18].

In this study, we carried out in-depth mining of second-generation sequencing transcriptomics data on liver cancer in The Cancer Genome Atlas (TCGA) database, modularized genes through differential expression analysis, compared module changes before and after liver cancer, and studied the corresponding genes in the module-enriched functional pathways to understand changes in gene regulation in liver cancer. In addition, we also compared the changes in gene regulation before and after liver cancer with the small-molecule compounds or drugs reported to interfere with the gene regulation in model species and selected the small-molecule compounds or drugs which caused reversed changes as the potential drugs for the treatment of cancer. Through these studies, we hope to develop systematic research and treatment programs for liver cancer in the future.

## 2. Materials and Methods

### 2.1. Gene Expression Data

The sample data (liver cancer) were obtained from TCGA database [19]. We collected RNA sequencing data (read count data) of all samples under the project ID of TCGA-LIHC. After excluding samples with low data quality (if the vial in the sample ID is B, it means formalin-fixed paraffin-embedded tissue, which has been proved to be ineffective for sequencing analysis, and this will be removed), we obtained a total of 421 liver cancer samples (50 normal samples and 371 cancer samples), in order to ensure the reliability of subsequent analysis. The significance of the difference between the cancer sample and the normal sample was compared, and the result was corrected by the Bonferoni method. The result showed that the difference between the groups was not significant (Supplementary Figure S1).

### 2.2. Dataset of Differentially Expressed Genes Affected by Drugs or Small Molecules

The dataset of differentially expressed genes with which drugs or small molecules could interfere was collected from Crowd Extracted Expression of Differential Signatures (CREEDS) (http://amp.pharm.mssm.edu/creeds) [20], which contained 8590 gene expression characteristics as affected by various small-molecule compounds or drugs.

### 2.3. Differential Expression Gene Extraction and Functional Enrichment Analysis

We applied a pipeline similar to Gao et al. [21]. Specifically, we used principal component analysis (PCA) to screen all samples of liver cancer and excluded the outliers to reduce sample disturbance. A total of 13 outliers were excluded. Subsequently, read counts were used to call differential expression genes between liver cancer and normal samples by using an R package DESeq2 [22] (adjusted *p* value <1*e*-5 was set as the threshold). We used ClueGO in Cytoscape (https://cytoscape.org/) to perform pathway enrichment analysis on the above differential gene expression genes [23]. The datasets used were from the GO, KEGG, and Reactome databases [24–26], and 0.05 was selected as the significance threshold.

### 2.4. Construction of Cancer and Normal Gene Coexpression Networks

We classified liver cancer samples and normal samples by hierarchical clustering provided by weighted gene correlation network analysis (WGCNA) and removed abnormal samples to construct a coexpression network [27]. The soft threshold was set as follows: normal group, 5 and liver cancer group, 5.

### 2.5. Analysis of Gene Regulatory Networks

Clusters of gene modules were obtained by WGCNA. The correlation of gene expression in each module was relatively high for genes belonging to the same regulator subnetwork and participating in the same functional regulation. We can understand the influence of the occurrence of liver cancer on the synergy between genes by comparing the number of clustering modules before and after liver cancer. We performed functional enrichment analysis on all modules gathered in the normal sample group (except the gray module; genes in the gray module were not related, or the correlation was not significant) and found functional pathways related to cancer regulation; these functional pathways were used as benchmarks. We compared the number of genes and the related changes in the modules enriched in these functional pathways in the corresponding liver cancer sample group to explore the internal regulatory relationship of related pathways before and after cancer and to understand the pathogenesis of cancer. In order to reveal the main functional pathways of each module, we use the ClueGO cyREST tool for functional enrichment analysis [28]. For gene modules with specific functions, we use DGCA (for differential gene correlation analysis, a comprehensive R package for differential gene correlation analysis) [29] to calculate the correlations between genes in the modules in the liver cancer group and the normal group. The correlation between genes in the final module is visualized by Cytoscape.

### 2.6. Analysis of Potential Applicability of Drugs

8590 drug perturbation-induced gene expression signatures collected in CREEDS were used in our analysis. Signatures from CREEDS were tanked using Fisher's exact test. We calculated the significance of overlap between the upregulation and downregulation of genes caused by drugs and the upregulated and downregulated genes in normal and cancer samples, respectively. The drugs were ranked on the basis of overlap observed between the genes induced by the drug and the differentially expressed genes in liver cancer.

## 3. Result

### 3.1. Differential Gene Analysis Identified Important HCC Genes Enriched in Many GO Terms

Results of PCA for all samples have been presented in Figure 1. DESeq2 was used after data processing. In liver cancer samples, we obtained 12,867 significantly differentially expressed genes compared to normal samples, with 4,533 upregulated and 8,334 downregulated genes.

Using the selected threshold screening (adjusted *p* value <1*e*-5), many significantly differentially expressed genes were detected. We decided to increase the screening criteria (adjusted *p* value ≤1*e*-5, base mean ≥ 10, and ∣ log2 fold change  | ≥1) according to the data distribution (Figure 2). We obtained 1,337 significantly differentially expressed genes, with 1,041 upregulated and 296 downregulated genes, compared with normal samples. Enrichment analysis results have been presented in Supplementary Table S1 and S2, including “*α*-adrenergic receptor activity” (GO:0004936), “adrenergic receptor activity” (GO:0004935), “epinephrine binding” (GO:0051379), “copper ions” (GO:0010273), “detoxification of inorganic compounds” (GO:0061687), “stress response to metal ions” (GO:0097501), “stress response to copper ion” (GO:0004935) in GO dataset, “metallothioneins bind metals” (R-HSA:5661231) [30], “RNA Polymerase I Promoter Opening” (R-HSA:73728) [31], and “SIRT1 negatively regulates rRNA expression” (R-HSA:427359) [32] in Reactome dataset, and “Neuroactive ligand-receptor interaction” (KEGG:04080), “Systemic lupus erythematosus” (KEGG:05322), and “Alcoholism” (KEGG:05034) in KEGG dataset. We have shown the top 10 pathways with the highest proportion of genes in the enrichment results of GO, KEGG, and Reactome (Figure 3).

### 3.2. HCC-Perturbed Coexpression Modules Identified by Gene Coexpression Submodule Analysis

We used the original data of differential gene analysis as the input data of WGCNA to conduct gene coexpression network analysis. The input data were divided into a normal group and a liver cancer group and analyzed separately to observe the synergistic effect between gene expression under different conditions. We removed the genes whose expression level was 0 in all samples, deleted the sample points of the partial segregation group according to the hierarchical clustering results of the samples (Figures 4(a) and 4(b)), and then performed coexpression network analysis. We finally obtained 84 gene modules in the liver cancer group and 45 gene modules in the normal group (Figures 4(c) and 4(d)). We found that in the liver cancer group, the number of submodules was significantly higher, the synergy of gene expression was lower, and the cell regulatory system tended to be disordered as compared with the normal group. The main functional pathways of each module revealed by functional enrichment analysis using ClueGO cyREST tool have been presented in Supplementary Table S3 and S4. There were 1,857 instances of annotation data for the submodules of the normal group and only 357 instances of annotation data for the submodules of the liver cancer group. Although the number of cancer submodules was higher, the corresponding functions of the modules were lower, which resulted in decline in system robustness.

In the analysis of gene coexpression network modules, compared with the normal group, the number of submodules in the liver cancer group is significantly increased, the synergy of gene expression is lower, and the cell regulation system tends to be chaotic. From this, we infer that the robustness of the system is reduced, cancerous cells cannot complete all the functions of normal cells, and the system function is mainly inclined to the direction of cell proliferation, for example.

In order to further understand how the coexpression module in liver cancer samples differed from the normal group, we compared the module sets of the two groups of samples. For each coexpression module in the liver cancer group, we selected a module in the normal group with the largest gene overlap corresponding to it. Total 84 coexpression network modules of liver cancer genes were mapped to 16 gene coexpression network modules from the normal group (Figure 5 and Supplementary Table S5 and S6).

In normal samples, the “pink” module gene was enriched in the adrenergic receptor activity, which was reported to be related to cancer [33]. In order to better represent the gene correlation within the modules, the “pink” module (637 genes) in the normal group was selected. We screened the gene pair correlation results calculated by DGCA (absolute value of correlation greater than 0.3, and *p* value <0.05) and plotted the network diagram (Figure 6). By analyzing the pathway enrichment of differentially expressed genes and comparing the changes in the coexpression module in liver cancer and normal tissues, we could understand the pathogenesis of cancer at the system level, which provides a reference for our drug therapy. By interfering with the expression of differentially expressed genes, we can reverse the differentially expressed genes in liver cancer cells and restore their normal expression levels.

### 3.3. Repositioning of Potential Drugs for Treating HCC

We used drug perturbation-induced gene expression signatures obtained from CREEDS to compare the genes whose expression was significantly different (*p* < 0.00001) in liver cancer and normal samples and calculated the intersection of the genes in each drug perturbation-induced gene expression signature with significantly different genes. The results of the comparison are shown in Supplementary Table S7, S8, and S9. The number of overlaps between the genes upregulated by drugs and the genes downregulated in liver cancer samples was sorted from large to small (*p* value <0.05, 3,576 results). The number of overlaps between the genes downregulated by drugs and the genes upregulated in liver cancer samples was also sorted from large to small (*p* value <0.05, 4 results). Under each screening condition, the top five drug or small-molecule perturbations were observed (duplicate tags were skipped) to see if they could treat liver cancer (Table 1). Most of the genes regulated by these drugs were significantly differentially expressed in gastric cancer (Table S4). This may provide new ideas and directions for the use of drugs.

## 4. Discussion

Analyzing the pathways enriched by the differential genes of human HCC (Supplementary TableS1 and S2), we found that there are many pathways related to *α*-adrenergic receptors, such as “*α*-adrenergic receptor activity” (GO:0004936), “adrenergic receptor activity” (GO:0004935), and “epinephrine binding” (GO:0051379). We suspect that this is obviously related to liver cancer. Through literature research, it has been reported that human HCC can cause profound changes in the hepatic *α*-adrenergic receptor signal transduction pathway and may lead to carbohydrate-related metabolic dysfunction and wasting syndrome in cancer patients [33]. There are also pathways related to metal ion metabolism, such as “detoxification pathway of copper ions” (GO:0010273), “detoxification of inorganic compounds” (GO:0061687), “stress response to metal ions” (GO:0097501), and “stress response to copper ion” (GO:0004935). The correlation between metal ions, such as copper, and liver cancer has also been reported [34]. Pathways that have been reported to be related to liver cancer also include “metallothioneins bind metals” (R-HSA:5661231) [30], “RNA Polymerase I Promoter Opening” (R-HSA:73728) [31], and “SIRT1 negatively regulates rRNA expression” (R-HSA:427359) [32]. These functional channels are all in our channel list, which also provides evidence to support the reliability of the data we analyze.

In the analysis of gene coexpression network modules, compared with the normal group, the number of submodules in the liver cancer group is significantly increased, the synergy of gene expression is lower, and the cell regulation system tends to be chaotic. From this, we infer that the robustness of the system is reduced. Cancerous cells cannot complete all the functions of normal cells, while the system functions are mainly tilted in a specific direction, such as cell proliferation.

During the screening of potential drugs, we discovered some potential small molecule drugs. The genes affected by these drugs overlap with the differentially expressed genes in liver cancer samples. And the genes whose expression is upregulated by drugs are significantly downregulated in liver cancer samples. Therefore, we believe that these drugs have the potential to affect gene expression in liver cancer samples and restore them to normal levels.

This paper proposes new ideas for the pathogenesis study and drug treatment for liver cancer. We used RNA sequencing read count data from liver cancer and normal samples as input files and gene expression characteristics induced by drug interference as reference files. By means of DESeq2 differential expression analysis, WGCNA gene coexpression network analysis, and comparative analysis of gene expression characteristics with drug effects, we explored the related pathway changes in liver cancer and obtained potential therapeutic drugs that highly matched the characteristics of alterations in gene expression due to liver cancer. This method is of great significance for systematically understanding the treatment mechanism, pathway change characteristics, and drug guidance for HCC. We will further analyze subnetwork modules, collect key gene sets related to cancer, and screen potential drugs for these key genes.

Because the liver cancer specimens collected by TCGA has come from multiple individuals and platforms, and the pathogenesis is different for each type of cancer, liver cancer contains multiple subtypes, which introduces certain errors and uncertainties in the analysis. In further studies, we will continue to improve this method and try to distinguish gene expression changes and pathway change characteristics of different subtypes. With the introduction and promotion of the concept of personalized medicine and the decreasing cost of next-generation sequencing, the proposed treatment method may become possible in the near future.

## Figures and Tables

**Figure 1:** Principal component analysis (PCA) of liver cancer samples. We can obtain the distribution of the samples on the principal component axis through the matrix decomposition method, which can be subsequently used to preprocess the sample data and remove outliers. (a) Original sample distribution; (b) filtered sample distribution; the red dot N indicates a normal sample point, and the blue dot T indicates a liver cancer sample point.

**Figure 2:** Data distribution plot for DESeq2 results. (a) Base mean frequency distribution of all genes and distribution of the mean for the gene's read counts in all samples; (b) log2 fold change frequency distribution of all genes and distribution of the mean value for the gene's fold change in all samples.

**Figure 3:** The top ten enrichment analysis results with the highest proportion of genes in GO, KEGG, and Reactome. The *x*-axis depicts the percentage of enriched differentially expressed genes in the corresponding pathway, and the *y*-axis presents the name of the pathway. GO enrichment analysis is on the top, whereas KEGG and Reactome enrichment analysis are merged below.

**Figure 4:** WGCNA analysis results. (a) Hierarchical clustering results of the normal group (cutoff = 2*e* − 6). (b) Hierarchical clustering results of the liver cancer group (cutoff = 3*e* − 6); both (a) and (b) select the branch with the most samples for subsequent analysis. (c) Normal group coexpression module (45 gene modules, except gray module). (d) Liver cancer sample coexpression module (84 gene modules, except gray module).

**Figure 5:** Correspondence map of cancer and normal gene modules. The *x*-axis is the gene coexpression module of the normal group, and the *y*-axis is the corresponding number of gene coexpression modules of each module in the liver cancer group.

**Figure 6:** Correlation of genes in the pink module in cancer and normal samples. (a) Normal group gene association analysis; (b) cancer group gene association analysis. Data with an absolute value of the correlation coefficient greater than 0.6 and a confidence level of less than 0.05 are shown. The red edges indicate a positive correlation, and the blue indicates a negative correlation. Most genes are positively related.

**Table 1:** List of potential therapeutic drugs for liver cancer.

Type	Drug/small molecule	Possible effect	Evidence (DOI)
a	Nutlin	Nutlin kills cancer cells via mitochondrial p53	10.4161/cc.8.11.8746 10.1124/mol.114.091603 10.1016/j.yexcr.2017.04.009
a	Paclitaxel|eribulin	Antimitotic agent	10.1159/000489067 10.1093/annonc/mdu435.56
a	17*β*-Estradiol	17*β*-Estradiol suppresses HCC cell proliferation and xenograft tumor development by inducing apoptosis	10.1371/journal.pone.0153863 10.1124/mol.63.6.1373
a	Enzalutamide	Inhibiting androgen; inhibition of tumor growth in response to androgen stimulation	10.1158/0008-5472.SABCS13-P2-09-05 10.1002/cncr.30336
b	6*α*-Methylprednisolone	Strong anti-inflammatory effect	10.1002/ddr.430020113 10.1111/nmo.12391
b	Histone deacetylase inhibitor	Effect on cell cycle regulation in hepatoma cells	10.7150/jca.34091 10.5392/IJoC.2012.8.4.074 10.1002/jcp.1087
b	4,4′-Diaminodiphenylmethane|inhibitor|(2Z,3Z)-bis{amino[(2-aminophenyl)sulfanyl]methylidene}butanedinitrile	Inhibitors of hepatocarcinogenesis	10.1093/carcin/2.10.1033
b	L-Proline residue|DNA damage-inducible transcript 3 protein	L-Proline-rich proteins and critical L-proline residues have a positive effect on the treatment of liver cancer	10.3892/mmr.1.4.459
b	Hemin	Inhibition of proliferation and induction of apoptosis of hepatoma cells	10.1196/annals.1299.055

^∗^Type “a” refers to the drugs that are used to improve the downregulated genes in liver cancer; type “b” refers to the drugs that are used to improve the upregulated genes in liver cancer. The drug label and possible mechanism of action are shown in the table, and literature support is provided.

## Data Availability

The data used to support the findings of this study are available from the corresponding author upon request.

## Supplementary Materials

Supplementary Materials Table S1: GO enrichment analysis. Table S2: KEGG and Reactome pathway enrichment analysis. Table S3: Module Path Enrichment Analysis. Table S4: Module Path Enrichment Analysis. Table S5: statistics list. Table S6: gene coexpression module. Table S7: comparison results of disturbed gene sets of drugs. Table S8: drugs increase the expression of downregulated genes. Table S9: drugs increase the expression of upregulated genes. Supplementary Figure S1: box plot of RNA read count data from cancer samples and normal samples.

## References

[1] Ryerson A. B., Eheman C. R., Altekruse S. F. (2016). Annual Report to the Nation on the Status of Cancer, 1975-2012, featuring the increasing incidence of liver cancer. *Cancer*.

[2] Wong M. C., Jiang J. Y., Goggins W. B. (2017). International incidence and mortality trends of liver cancer: a global profile. *Scientific Reports*.

[3] Xu X.-R., Huang J., Xu Z.-G. (2001). Insight into hepatocellular carcinogenesis at transcriptome level by comparing gene expression profiles of hepatocellular carcinoma with those of corresponding noncancerous liver. *Proceedings of the National Academy of Sciences*.

[4] Anwanwan D., Singh S. K., Singh S., Saikam V., Singh R. (2020). Challenges in liver cancer and possible treatment approaches. *Biochimica et Biophysica Acta (BBA)-Reviews on Cancer*.

[5] Cai Y., Yang J., Huang T., Wang M. W. (2021). Editorial: computational methods in predicting complex disease associated genes and environmental factors. *Frontiers in Genetics*.

[6] Liu H., Qiu C., Wang B. (2021). Evaluating DNA methylation, gene expression, somatic mutation, and their combinations in inferring tumor tissue-of-origin. *Frontiers in Cell and Development Biology*.

[7] He B., Dai C., Lang J. (2020). A machine learning framework to trace tumor tissue-of-origin of 13 types of cancer based on DNA somatic mutation. *Biochimica et Biophysica Acta (BBA) - Molecular Basis of Disease*.

[8] He B., Lang J., Wang B. (2020). TOOme: a novel computational framework to infer cancer tissue-of-origin by integrating both gene mutation and expression. *Frontiers in Bioengineering and Biotechnology*.

[9] Liu C., Wei D., Xiang J. (2020). An improved anticancer drug-response prediction based on an ensemble method integrating matrix completion and ridge regression. *Mol Ther Nucleic Acids*.

[10] Fu J., Wang H. (2018). Precision diagnosis and treatment of liver cancer in China. *Cancer Letters*.

[11] Sun J., Wei Q., Zhou Y., Wang J., Liu Q., Xu H. (2017). A systematic analysis of FDA-approved anticancer drugs. *BMC Systems Biology*.

[12] Chen E. Y., Raghunathan V., Prasad V. (2019). An overview of cancer drugs approved by the US Food and Drug Administration based on the surrogate end point of response rate. *JAMA Internal Medicine*.

[13] Liu X., Yang J., Zhang Y. (2016). A systematic study on drug-response associated genes using baseline gene expressions of the Cancer Cell Line Encyclopedia. *Scientific Reports*.

[14] Yang J., Peng S., Zhang B. (2020). Human geroprotector discovery by targeting the converging subnetworks of aging and age-related diseases. *Geroscience*.

[15] Xu X., Long H., Xi B. (2019). Molecular network-based drug prediction in thyroid cancer. *International Journal of Molecular Sciences*.

[16] Yang J., Huang T., Song W. M. (2016). Discover the network underlying the connections between aging and age-related diseases. *Scientific Reports*.

[17] Li T., Huang T., Guo C. (2021). Genomic variation, origin tracing, and vaccine development of SARS-CoV-2: A systematic review. *Innovation (N Y)*.

[18] Tang X., Cai L., Meng Y., Xu J., Lu C., Yang J. (2021). Indicator regularized non-negative matrix factorization method-based drug repurposing for COVID-19. *Frontiers in Immunology*.

[19] Tomczak K., Czerwińska P., Wiznerowicz M. (2015). Review The Cancer Genome Atlas (TCGA): an immeasurable source of knowledge. *Contemporary oncology*.

[20] Wang Z., Monteiro C. D., Jagodnik K. M. (2016). Extraction and analysis of signatures from the Gene Expression Omnibus by the crowd. *Nature Communications*.

[21] Gao W., Yang J., Zhuo C. (2020). A pipeline to call multilevel expression changes between cancer and normal tissues and its applications in repurposing drugs effective for gastric cancer. *BioMed Research International*.

[22] Love M. I., Huber W., Anders S. (2014). Moderated estimation of fold change and dispersion for RNA-seq data with DESeq2. *Genome biology*.

[23] Bindea G., Mlecnik B., Hackl H. (2009). ClueGO: a Cytoscape plug-in to decipher functionally grouped gene ontology and pathway annotation networks. *Bioinformatics*.

[24] Consortium G. O. (2004). The Gene Ontology (GO) database and informatics resource. *Nucleic acids research*.

[25] Kanehisa M., Goto S. (2000). KEGG: kyoto encyclopedia of genes and genomes. *Nucleic Acids Research*.

[26] Croft D., O’Kelly G., Wu G. (2011). Reactome: a database of reactions, pathways and biological processes. *Nucleic acids research*.

[27] Langfelder P., Horvath S. (2008). WGCNA: an R package for weighted correlation network analysis. *BMC bioinformatics*.

[28] Mlecnik B., Galon J., Bindea G. (2019). Automated exploration of gene ontology term and pathway networks with ClueGO-REST. *Bioinformatics*.

[29] McKenzie A. T., Katsyv I., Song W.-M., Wang M., Zhang B. (2016). DGCA: a comprehensive R package for differential gene correlation analysis. *BMC systems biology*.

[30] Cherian M. G., Jayasurya A., Bay B.-H. (2003). Metallothioneins in human tumors and potential roles in carcinogenesis. *Mutation Research/Fundamental and Molecular Mechanisms of Mutagenesis*.

[31] Bhoola K. D., Misso N. L., Naran A., Thompson P. J. (2007). Current status of tissue kallikrein inhibitors: importance in cancer. *Current Opinion in Investigational Drugs*.

[32] Koga T., Suico M. A., Shimasaki S. (2015). Endoplasmic reticulum (ER) stress induces sirtuin 1 (SIRT1) expression via the PI3K-Akt-GSK3*β* signaling pathway and promotes hepatocellular injury. *Journal of Biological Chemistry*.

[33] Kassahun W. T., Günl B., Jonas S., Ungemach F. R., Abraham G. (2011). Altered liver *α*_1_-adrenoceptor density and phospholipase C activity in the human hepatocellular carcinoma. *European Journal of Pharmacology*.

[34] Mori M., Hattori A., Sawaki M. (1994). The LEC rat: a model for human hepatitis, liver cancer, and much more. *The American journal of pathology*.

